# Effect of Lianhuaqingwen Capsules on Airway Inflammation in Patients with Acute Exacerbation of Chronic Obstructive Pulmonary Disease

**DOI:** 10.1155/2014/637969

**Published:** 2014-05-25

**Authors:** Liang Dong, Jing-wen Xia, Yi Gong, Zhen Chen, Hai-hua Yang, Jing Zhang, Jian He, Xiao-dong Chen

**Affiliations:** Department of Pneumology, Huashan Hospital, Fudan University, No. 12 Wulumuqi Zhong Road, Shanghai 200040, China

## Abstract

Chronic obstructive pulmonary disease (COPD) is characterized by a chronic inflammatory response that is worsened by acute exacerbations. Lianhuaqingwen (LHQW) has anti-inflammatory and immune regulatory functions and may inhibit the airway inflammation that occurs during an acute exacerbation of COPD. In this study, 100 participants were recruited and randomly assigned, 1 : 1, to the LHQW and the conventional groups, which were treated, respectively, with LHQW capsules and conventional Western medicine or only conventional Western medicine. The scores of the CAT scale and levels of inflammatory cytokines in blood and sputum were measured during treatment. In addition, subjects were subdivided into high-risk and low-risk subgroups. The CAT scores in the LHQW group and high-risk subgroup were clearly improved from the 5th day, but the other groups improved only after treatment was completed. Expression levels of IL-8, TNF-**α**, IL-17, and IL-23 in the sputum and of IL-8 and IL-17 in the blood were significantly decreased after treatment, and similar results were found in subgroups. These data suggested that LHQW capsules can accelerate the improvement of AECOPD patients, especially for the high-risk subgroup, and the mechanism of action may be related to the decreased release of inflammatory mediators.

## 1. Introduction

Chronic obstructive pulmonary disease (COPD) is a persistent disease characterized by limited airflow and disease progression that has a high morbidity and mortality worldwide [1]. In 2011, a nationwide epidemiological survey in the USA found that the prevalence of COPD was 6.3% overall and was 11.6% in the population older than 65 years [2]. Gong et al. [3] carried out an epidemiological survey of the population over 60 years of age residing in Shanghai urban areas; the results showed that the prevalence rate of COPD was 14.61%, which is an increase of 8.3% compared with five years ago.

Acute exacerbation of chronic obstructive pulmonary disease (AECOPD) is an important event in the natural progression of COPD. AECOPD can aggravate the symptoms of chronic airway inflammation associated with airway remodeling in COPD patients, accelerate the progression of airway obstruction, produce a rapid decline in lung function and quality of life, increase the rates of complications, admissions, and mortality [4, 5], and have a great impact on individual and societal economic burdens [6, 7]. AECOPD especially affects patients with moderate to severe COPD, who are most vulnerable to its effects [8]. Studies have shown that infections with bacteria, viruses, and atypical pathogens are the most important factors that induce AECOPD [9]; mixed infections of bacteria and viruses are common in AECOPD [10, 11]. Bacterial colonization occurs in the airways of stable COPD patients; an increase in the bacterial load to a certain level or the acquisition of a new virulent strain can cause an acute exacerbation, resulting in severe inflammation [12, 13]. The Global Initiative for Control and Prevention of Chronic Obstructive Pulmonary Disease (GOLD) [1] recommends hormones, antibiotics, bronchodilators, and symptomatic and supportive therapy as the primary treatment program for AECOPD. However, this program has not produced a satisfactory effect, and large doses of these recommended drugs may increase the risk of infection [14]; thus, we need to evaluate more effective drugs to treat AECOPD.

Lianhuaqingwen (LHQW) is a compounded Chinese herbal medicine that is produced by addition and reduction of combined Yinqiao powders and Maxing Shigan decoction, which has multiple therapeutic targets and comprehensive therapeutic action [15]. Mo et al. [16] gave LHQW capsules to patients with human influenza A virus infection for different time periods and found that it affects various parts of or inhibits human influenza A virus infection through several mechanisms, including prevention of virus adsorption, inhibition of replication and proliferation after viral adsorption, and having a direct antivirus effect. The experimental studies performed by China Academy of Traditional Chinese Medicine showed a definite antibacterial action of LHQW, which could disrupt bacterial biofilms, significantly inhibit the number of viable cells at the intramembrane, and have bacterial resistance properties. The Pharmacology of Traditional Chinese Medicine, Hebei Medical University, found that LHQW had inhibiting effects on* Staphylococcus aureus*, alpha- and beta-hemolytic* Streptococcus*,* pneumococcus*,* Haemophilus*, and influenza. Li [17] analyzed 136 cases with influenza complicated with bronchial pneumonia and found that patients who received LHQW capsules had more symptom improvement than did those in the control group. These findings indicated that LHQW was effective for concurrent viral and bacterial infections. Guo et al. [18] investigated the influenza virus infection of blood T lymphocyte subsets in mice and found that LHQW had regulatory functions on cellular immunity. The above studies suggested that LHQW can be used to treat AECOPD due to its anti-infective and immunomodulatory effects. In animal experiments, our research group [19] found that LHQW capsules could clearly reduce the levels of IL-8 and TNF-*α* in serum, lung tissue, and bronchial lavage fluid of COPD rats (*P* < 0.01), and we confirmed its ability to suppress airway inflammation in COPD rats.

Therefore, we intend to further explore the effect of LHQW capsules on the airway inflammation of patients with AECOPD, to investigate its mechanism of action by studying innate immune factors, such as interleukin-8 (IL-8) and tumor necrosis factor-*α* (TNF-*α*), and acquired immune factors, such as interleukin-17 (IL-17) and interleukin-23 (IL-23), to explore the application value of LHQW for treating AECOPD, and to provide an additional, new choice for treating AECOPD with traditional Chinese medicine (TCM).

## 2. Materials and Methods

### 2.1. Participants

From January 2012 to January 2013, 100 subjects were enrolled from the AECOPD inpatients and outpatients at our hospital; these patients included 86 males and 14 females and had a mean ± SD age of 71.50 ± 10.17 years. All of the subjects were diagnosed with AECOPD according to the GOLD diagnosis and treatment guideline (2011 edition) [1] and had an adequate understanding of the procedures and purpose of this trial and signed the informed consent form.

The exclusion criteria were any one of the following conditions: (1) age <50 or >85 years old; (2) blood gas analysis indicating respiratory failure (PaO_2_ < 60 mmHg and/or PaCO_2_ > 50 mmHg when breathing quietly without oxygen at sea level) and the patient required mechanical ventilation; (3) coexisting serious primary diseases (heart, cerebrovascular, hepatic, renal, or hematologic disease), impaired immune function (including cancer and autoimmune diseases), psychopathology, pregnancy, or breast feeding women; (4) upper or lower respiratory tract infection in the two months before the enrollment date; (5) use of TCM to treat the disease within 36 hours of enrollment; and (6) known allergy to the composition of LHQW, to food, or to more than two drugs.

### 2.2. Materials

The main components of LHQW are Forsythiae Fructus (255 g), Ephedrae Herba (honey-fried) (85 g), Lonicerae Japonicae Flos (255 g), Isatidis Radix (255 g), Dryopteris Crassirhizomatis Rhizoma (255 g), menthol (7.5 g), Gypsum Fibrosum (255 g), Pogostemonis Herba (85 g), Rhodiolae Crenulatae Radix et Rhizoma (85 g), Houttuyniae Herba (255 g), Rhei Radix et Rhizoma (51 g), Armeniacae Semen Amarum (stir-baked) (85 g), and* Glycyrrhizae Radix et Rhizoma* (85 g), and the excipient is starch. These LHQW capsules were donated by Yiling Pharmaceutical Inc. (Shijiazhuang, China), TCM Quasiword, Z20040063; product batch, 111010; product specifications, 0.35 g per capsule.

### 2.3. Study Design

All of the participants were randomly assigned to either the LHQW treatment group or the conventional treatment group (the LHQW group and the conventional group, resp.) in a 1 : 1 ratio; 50 patients were allocated to each group. Subjects in both groups were given conventional treatment for AECOPD (inhaled medications, salmeterol/fluticasone, 250/50 *μ*g; bronchodilators, theophylline; expectorant antispasmodic agent, ambroxol; antibacterial agents, *β*-lactams, if allergic to *β*-lactams then fluoroquinolones were given; and controlled oxygen therapy). The patients in the LHQW group were also administered LHQW capsules orally (1.4 g per time, 3 times per day, for 7 days).

We recorded age, gender, body mass index (BMI), allergy and disease history, use of TCM and other medicines, exacerbation history (in the last year), blood test results, chest X-ray results, blood gas analysis results, and pulmonary function tests at study enrollment. Smoking history, duration of COPD (years since first diagnosis of COPD), COPD assessment test (CAT), and blood and sputum samples were obtained at admission. Participants were assessed by the CAT on the 3rd and 5th days of treatment. At the end of the treatment period, day 7, all subjects were asked to return for another CAT, blood gas analyses, pulmonary function tests, and blood and sputum samples. The study protocol was approved by the local institutional ethics committee (Huashan Hospital, Fudan University, Shanghai, China, 2011, clinical trial review number 198), registered on the Chinese Clinical Trial Registry (ChiCTR-TRC-13003240).

### 2.4. Induced Sputum Samples

All participants were instructed to rinse their mouth and throat and to expectorate deeply. Sputum samples were diluted with an equal volume of 0.1% dithiothreitol (DTT) and incubated for 15 min at 37°C. Within two hours, the solution was centrifuged at 3,000 rpm for 10 min, if the sputum specimen was considered to be adequate (>25 neutrophils and <10 squamous epithelial cells per low power field). After centrifugation, the supernatants were harvested and stored at −80°C until needed.

If no sputum was produced after deep expectoration, we performed sputum induction (SI) using an adapted protocol by Sutherland et al. [20] and Bathoorn et al. [21] for use in AECOPD patients. Briefly, immediately before the procedure, the baseline FEV_1_ was recorded, and an inhaled dose of salbutamol (200 *μ*g) was given, followed by spirometry 10 min later. Then, SI was performed. The subjects with an FEV_1_% Pred that was <50% inhaled a nonbuffered isotonic saline solution (0.9% NaCl), and all of the other patients inhaled a hypertonic saline solution (3% NaCl). FEV_1_ was monitored every 2 minutes. If the FEV_1_ decreased by ≥20% or if symptoms appeared difficult to tolerate, the SI was completely stopped. If the FEV_1_ decreased by 10 to 20%, the participants received salbutamol (200 *μ*g), and we measured FEV_1_ again 10 min later. If the decrease in FEV_1_ was still >10%, the SI was stopped. After each step, the subjects were asked to expectorate sputum. If the sputum volume produced after 12 min was insufficient, we increased the NaCl concentration of the saline solution to 4.5% for the last time. To ensure safety, the oxygen saturation of all subjects was monitored throughout the process until the SI was finished and until the FEV_1_ was >90% of the baseline post-salbutamol FEV_1_ value.

### 2.5. Serum Samples

10 mL of venous blood was drawn into plastic tubes containing ethylenediamine tetraacetic acid and was centrifuged at 3,000 rpm for 10 min within an hour. The serum samples were collected and stored at −80°C until analysis.

### 2.6. Quantification of Inflammatory Mediators

The levels of IL-8, TNF-*α*, IL-17, and IL-23 in serum and sputum supernatants were quantified by commercially available enzyme-linked immunosorbent assay (ELISA), according to manufacturer's protocols (Senxiong Biotech, Shanghai, China).

### 2.7. Statistical Analysis

Windows SPSS19.0 statistical software was used. Normally distributed data were expressed as mean ± standard deviation (mean ± SD). The independent samples *t*-test was used to compare two groups, and the univariate analysis of variance (one-way ANOVA) was used to compare means of > two groups. If a statistically significant difference was found, the least significant difference (LSD) method was used for the comparison of two groups. *P* < 0.05 was considered to be a significant difference.

## 3. Results 

### 3.1. Clinical Characteristics of Participants

A total of 146 subjects were screened for eligibility; 46 subjects could not be included. The main reason for noninclusion was not meeting the inclusion criteria mainly due to the subject being complicated with respiratory failure (see Figure 1). 100 AECOPD subjects were randomized within two groups: 50 in the LHQW group and 50 in the conventional group. No significant difference was found in age, gender, body mass index (BMI), smoking history, lung function tests, and blood gas analyses between the two groups (*P* ≥ 0.05) (see Table 1). According to assessment criteria for acute exacerbation in the GOLD guideline, participants in the LHQW and conventional groups were categorized into low-risk subgroup (COPD comprehensive assessment group A-B) and high-risk subgroup (COPD comprehensive assessment group C-D) (see Table 2). The frequency of the subgroups was compared between treatments.

### 3.2. Changes in Clinical Manifestations after Treatment

We used the CAT scale to assess the symptoms and signs of AECOPD patients in each treatment group and subgroup. Before treatment, the mean CAT scores were 23.7 ± 8.17 points and 23.89 ± 7.9 points in the LHQW and conventional groups; these scores were not significantly different (*P* > 0.05). After 7 days of therapy, the mean scores decreased to 18.24 ± 7.55 and 18.89 ± 8.19 points, respectively; both scores clearly improved after treatment (*P* < 0.01). Furthermore, during treatment, we found that the scores were not different on the 3rd day, but on the 5th day, the mean score was 19.5 ± 7.61 points in the LHQW group, which was dramatically decreased relative to the pretreatment value (*P* < 0.01), while the conventional group mean score was 20.91 ± 8.05 points, which still was not significantly different (see Figure 2(a)). We analyzed the subgroups; in the high-risk subgroup, we found a pattern of results similar to that described above (see Figure 2(b)). However, in the low-risk subgroup, symptoms were significantly improved only after 7 days of treatment, and the two groups did not differ significantly during treatment (see Figure 2(c)).

### 3.3. Changes in the Sputum Levels of Cytokines after Treatment

In the LHQW group, the mean levels of IL-8, TNF-*α*, IL-17, and IL-23 in the sputum were 578.32 ± 200.27 pg/mL, 52.87 ± 25.26 pg/mL, 49.51 ± 22.42 pg/mL, and 27.02 ± 11.45 pg/mL before treatment and clearly decreased to 473.36 ± 200.55 pg/mL, 36.78 ± 20.17 pg/mL, 35.68 ± 17.66 pg/mL, and 19.09 ± 8.87 pg/mL, respectively, after treatment with LHQW capsules (see Figure 3(a), *P* < 0.05, and Figures 3(b), 3(c), and 3(d), *P* < 0.01). However, no significant differences in these cytokines levels were observed in the conventional group after treatment. Obviously (see Table 3), it was found that IL-8, TNF-*α*, and IL-17 decreased after treatment in the high-risk subgroup (*P* < 0.05), and TNF-*α*, IL-17, and IL-23 decreased after treatment in the low-risk subgroup (*P* < 0.05, *P* < 0.01). In contrast, in the conventional subgroups, the cytokines levels did not decrease significantly after treatment.

### 3.4. Changes in the Blood Levels of Cytokines after Treatment

The before and after treatment comparison showed that the level of blood IL-8 decreased after LHQW treatment (Figure 4(a), *P* < 0.05). The blood level of IL-17 was 111.62 ± 38.09 pg/mL before treatment and decreased to 93.16 ± 29.44 pg/mL after treatment (Figure 4(c),  *P* < 0.01). In the LHQW group, we found that blood levels of TNF-*α* and IL-23 had a declining trend during treatment that was not statistically significantly different (see Figures 4(b) and 4(d)); however, in the conventional group, we found that none of the cytokine levels changed significantly. In the LHQW subgroups (see Table 4), we found that IL-8 blood levels decreased in the low-risk subgroup after treatment (*P* < 0.05) and had a downward trend in the high-risk subgroup, but IL-17 blood levels decreased significantly in both the low-risk and high-risk subgroups (*P* < 0.05). In contrast, no statistically significant changes in cytokine blood levels were found in the conventional subgroups.

## 4. Discussions

Chinese medicine attributes COPD to cough, asthma, gasp syndrome, phlegm and retained fluid, lung heat, lung inflation, and other causes. Explanations for this pathology are that chronic illness results in a deficiency syndrome in the lung, phlegm is blocked in the body, and exogenous pathogenic factors can lead to onset or worsening of the disease. According to the* General Treatise on the Cause and Symptoms of Disease*, “when there was more gas in lung, the disease would be caused, and the lung distension was found.” Most scholars believe that COPD is a deficiency syndrome of the human body but it manifests as asthenic syndrome. COPD is usually caused by prolonged exposure to a variety of exogenous pathogenic factors; invasion by these factors leads to impaired lung qi and lung deficiency, and thus the lung, spleen, and kidney are impaired, and yin-yang disharmony occurs. It involves deficiency of lung, spleen, and kidney; deficiency of gas, yin, and yang; and insufficiency of pectoral qi; the inability to promote blood circulation results in dysfunction of qi and blood in internal organs, blood stasis, and sputum-blocked airways. Phlegm stagnation persists for a long time; therefore, the disease course is prolonged. TCM therapy for COPD always follows the principles of eliminating evil and strengthening the bodily constitution.

LHQW has anti-inflammatory and immune regulatory functions that are derived from the components of TCM. Among these components, Forsythiae Fructus, Menthol, and Ephedrae Herba can disperse the cold; Gypsum Fibrosum, Lonicerae Japonicae Flos, and Isatidis Radix can clear internal qi and endogenous heat; Armeniacae Semen Amarum and Houttuyniae Herba can detoxify and remove carbuncles; Rhei Radix et Rhizoma clears hollow viscera and lung heat; and Rhodiolae crenulatae Radix et Rhizoma has the function of tonifying qi and yin, regulating immunity, strengthening body resistance, and eliminating evil. In this study, we analyzed 100 patients with AECOPD who were treated either with LHQW and conventional Western medicine or with only conventional Western medicine. We measured subjects' clinical symptoms and signs and the levels of IL-8, TNF-*α*, IL-17, and IL-23 in the blood and sputum before and after treatment and thereby investigated the effects of LHQW on airway inflammation of AECOPD and its possible mechanism of action.

The aims of AECOPD treatment are to reduce the current clinical manifestations of the acute exacerbation and to prevent future exacerbations. In this study, we used the CAT scale to assess patient's clinical manifestations. The CAT scale is a simple quality of life rating scale developed by Jones PW in 2009 that is based on the St. George's Respiratory Questionnaire (SGRQ). This scale correlates well with SGRQ [22], but its content is relatively simple; it comprises 8 questions that can be answered within 3 min. We found that patients in both the LHQW and the conventional groups improved significantly after 7 days of treatment. The CAT scores were decreased from the 5th day in the LHQW group but not in the conventional group. To better assess the value of LHQW, we divided the patients into two subgroups (low-risk subgroup and high-risk subgroup), which were analyzed and compared. In the high-risk subgroup, we found the same outcomes as above; in the low-risk subgroup, symptoms were not improved until the 7th day of treatment. However, no significant difference was found between the two treatment groups during the process. This study indicated that LHQW can accelerate the improvement of clinical symptoms and signs for AECOPD patients, especially for high-risk subgroups, and its effectiveness may be greater with early application.

IL-8 and TNF-*α* both are important mediators of AECOPD [23, 24]. TNF-*α* is an early inflammation initiation factor [25] and can activate endothelial cells, stimulate the relative expression of adhesion molecules, and induce neutrophils to migrate and release IL-8, which has a strong chemotactic effect on leukocytes, and can enhance neutrophil function, induce neutrophil degranulation, and facilitate more TNF-*α* expression [26]. During an acute exacerbation of COPD, the respiratory tract is infected with viruses and/or bacteria. Therefore, exposure to certain microbial antigens or metabolites, such as LPS or endotoxin, can activate macrophages and neutrophils and thereby further increase inflammatory cytokines, such as IL-8 and TNF-*α*. Such increases lead to systemic and local chronic airway inflammation [27–29], a condition that causes COPD progression. In this study, the expression levels of both IL-8 and TNF-*α* in the sputum decreased in the LHQW group after treatment, but only the IL-8 levels in the blood decreased significantly after treatment. Further subgroup analysis showed that, in the LHQW group, the sputum levels of IL-8 decreased significantly in the high-risk subgroup after treatment (see Table 3), whereas the blood levels of IL-8 declined significantly in the low-risk subgroup (see Table 4). These findings may be explained by higher levels of systemic inflammation in COPD patients in the high-risk subgroup and by more marked airway inflammation during an acute exacerbation. In both subgroups, the TNF-*α* levels declined in the sputum, although the decline in TNF-*α* blood levels was not significant. Almansa et al. [30] and Pinto-Plata et al. [31] measured various inflammatory cytokines before and after treatment of AECOPD. Their results showed that serum IL-8 expression was significantly reduced but that TNF-*α* did not change significantly; these findings are consistent with our results. Groenewegen et al. [32] compared the expression of two TNF-*α* receptors, TNFR55 and TNFR75, before and after treatment. They found that these two receptors increased before treatment; TNFR75 rapidly decreased by the first day after treatment; TNFR55 was not changed significantly by the first, 4th, and 8th days after treatment, and both receptors recovered to normal levels 1 month later. Therefore, we considered that TNF-*α* receptor might be expressed differently in different populations, which partly explained why there is no TNF-*α* expression in the blood.

COPD is not only a chronic inflammatory disease [33] but also an autoimmune disease [34]. IL-17 can regulate innate immune responses by participating in the adaptive immune response [35], which requires IL-23 for differentiation and maturation [36]. Di Stefano et al. [37] obtained bronchial mucosa biopsies from patients with stable COPD and found that levels of IL-17A and IL-22 were increased in the bronchial mucosa and that IL-22 and IL-23 were increased in the bronchial epithelial. Zhang et al. [38] also found that CD4+ IL17+ cells expression levels were higher in the alveolar wall of patients with COPD than those in healthy individuals, and this expression was positively correlated with airway obstruction, which indicated that IL-17 played an important role in COPD occurrence and development [39]. When COPD exacerbates, antigen-presenting cells (e.g., dendritic cells) secrete IL-23, which combines with IL-23 receptor at the surface of Th17 cells, inducing secretion of IL-17 and regulating the inflammatory response [40, 41]. Our research found that expression of IL-17 was clearly decreased in the blood and sputum of patients with AECOPD in the LHQW group and in both LHQW subgroups after treatment but that IL-23 was significantly decreased only in the sputum in the LHQW treatment group and its low-risk subgroup; no significant change was found in the conventional group (see Tables 3 and 4). During this study, we thought that LHQW may play a role in immune regulation by IL-17, but whether this role is limited to acute exacerbation or also functions during the stable phase is still unclear. Notably, we found that the changes in IL-17 and IL-23 appeared to have different patterns. This phenomenon may be caused by normal pathophysiological conditions, changes in IL-17 and IL-23 at different stages of treatment, short length of follow-up, or insufficient sample size, and it needs further exploration.

## 5. Conclusions

In conclusion, the findings of this study support the hypotheses that this compounded traditional Chinese medicine, LHQW capsules, (1) could accelerate improvement of the clinical symptoms and signs of AECOPD, especially in patients in the high-risk subgroup; (2) play an important role in treating AECOPD; and (3) may be more effective if applied sooner. The mechanisms of action of LHQW may be reduced systemic and airway inflammation by regulation of the inherent and acquired immune systems through inhibition of the release of the corresponding inflammatory factors. However, the treatment program of herbal medicines in treating COPD is acknowledged to still lack, and we need to further study the mechanisms and effects of LHQW.

## Figures and Tables

**Figure 1:** The patients flow chart.

**Figure 2:** Changes in the CAT scores for the LHQW and conventional groups before and after treatment. The CAT scores were recorded before treatment and on the 3rd, 5th, and 7th days. (a) Changes in CAT score for the treatment groups; (b) changes in CAT score for the high-risk subgroups; (c) changes in CAT score for the low-risk subgroups. Each data point represents the mean score (*n* = 50). *P < 0.05 compared with the pretreatment CAT score in the LHQW group, **P < 0.01 compared with the pretreatment CAT score in the LHQW group, ^#^ *P* < 0.05 compared with the pretreatment CAT score in the conventional group, and ^##^ *P* < 0.01 compared with the pretreatment CAT score in the conventional group.

**Figure 3:** IL-8, TNF-*α*, IL-17, and IL-23 levels in the sputum of the LHQW and conventional groups before and after treatment. (a) Levels of IL-8 (pg/mL); (b) levels of TNF-*α* (pg/mL); (c) levels of IL-17 (pg/mL); and (d) levels of IL-23 (pg/mL). Each bar indicates the mean ± SD value (SD: standard deviation, *n* = 50). *P < 0.05 compared with values before treatment and **P < 0.01 compared with values before treatment.

**Figure 4:** IL-8, TNF-*α*, IL-17, and IL-23 levels in the blood of patients in the LHQW and conventional groups before and after treatment. (a) Levels of IL-8 (pg/mL); (b) levels of TNF-*α* (pg/mL); (c) levels of IL-17 (pg/mL); and (d) levels of IL-23 (pg/mL). Each bar indicates the mean ± SD (SD: standard deviation, *n* = 50). *P < 0.05 compared with values before treatment and **P < 0.01 compared with values before treatment.

**Table 1:** Baseline characteristics of participants in both study groups.

	LHQW group (*n* = 50)	Conventional group (*n* = 50)	Statistical significance
Age, years (mean ± SD)	70.62 ± 10.19	72.60 ± 9.54	NS
Gender (male, %)	44 (88%)	42 (84%)	NS
BMI, Kg/m^2^ (mean ± SD)	23.35 ± 3.66	22.90 ± 3.66	NS
Smoking history, pack years (mean ± SD)	765.19 ± 545.25	795.71 ± 500.39	NS
FEV_1_%Pred, % (mean ± SD)	50.32 ± 16.05	47.60 ± 18.78	NS
FEV_1_/FVC, % (mean ± SD)	65.84 ± 11.10	62.20 ± 18.43	NS
PO_2_, mmHg (mean ± SD)	76.64 ± 15.22	72.91 ± 16.58	NS
PCO_2_, mmHg (mean ± SD)	43.40 ± 5.53	45.35 ± 8.70	NS
SPO_2_, % (mean ± SD)	94.55 ± 10.92	91.04 ± 9.56	NS

NS: nonsignificant difference between the two groups, *P* value ≥0.05. SD: standard deviation, BMI: body mass index = weight (kg)/height^2^ (m^2^), FEV_1_%Pred: forced expiration volume in one second %predicted FEV_1_, FEV_1_/FVC: forced expiratory volume in one second/forced vital capacity, PO_2_: partial pressure of oxygen, PCO_2_: partial pressure of carbon dioxide, SPO_2_: oxygen saturation, 1 mmHg = 0.133 kpa.

**Table 2:** Comprehensive assessment of COPD participants.

Group	LHQW group (*n* = 50)	Conventional group (*n* = 50)	Statistical significance
Low-risk subgroups (A-B groups)	25	20	NS
High-risk subgroups (C-D groups)	25	30	NS

NS: nonsignificant difference between the two groups, *P* value ≥0.05.

**Table 3:** Levels of IL-8, TNF-*α*, IL-17, and IL-23 in the sputum of the LHQW group, the conventional group, and subgroups before and after treatment.

		Total		High-risk subgroups		Low-risk subgroups	
		LHQW group (*n* = 50)	Conventional group (*n* = 50)	LHQW group (*n* = 25)	Conventional group (*n* = 30)	LHQW group (*n* = 25)	Conventional group (*n* = 20)
IL-8	Before treatment (mean ± SD, pg/mL)	578.32 ± 200.27	582.70 ± 185.18	651.14 ± 159.52	636.89 ± 163.70	502.02 ± 213.45	525.44 ± 177.32
	After treatment (mean ± SD, pg/mL)	473.36 ± 200.55*	545.02 ± 168.19	547.01 ± 192.51*	587.04 ± 158.16	396.21 ± 182.58	493.09 ± 169.87
	*P* value	0.01	0.318	0.042	0.261	0.070	0.586

TNF-*α*	Before treatment (mean ± SD, pg/mL)	52.87 ± 25.26	53.80 ± 24.96	52.83 ± 25.64	58.17 ± 26.94	52.92 ± 25.48	48.08 ± 21.59
	After treatment (mean ± SD, pg/mL)	36.78 ± 20.17**	43.42 ± 21.57*	37.02 ± 21.05*	46.61 ± 19.98	36.54 ± 19.73*	39.76 ± 23.72
	*P* value	0.001	0.026	0.029	0.065	0.022	0.251

IL-17	Before treatment (mean ± SD, pg/mL)	49.51 ± 22.42	49.70 ± 23.87	50.93 ± 23.45	52.16 ± 25.09	48.03 ± 21.77	47.48 ± 22.12
	After treatment (mean ± SD, pg/mL)	35.68 ± 17.66**	42.84 ± 20.49	39.93 ± 16.99*	43.83 ± 20.59	34.39 ± 18.67*	42.29 ± 20.97
	*P* value	0.003	0.110	0.037	0.151	0.038	0.434

IL-23	Before treatment (mean ± SD, pg/mL)	27.02 ± 11.45	25.87 ± 12.04	27.53 ± 12.55	28.77 ± 13.31	26.49 ± 10.46	22.19 ± 8.94
	After treatment (mean ± SD, pg/mL)	19.09 ± 8.87**	21.14 ± 10.42*	20.32 ± 10.42	24.24 ± 11.78	17.79 ± 6.93**	17.24 ± 6.13
	*P* value	0.001	0.03	0.051	0.158	0.001	0.063

SD: standard deviation, *P < 0.05 compared with values before treatment, **P < 0.01 compared with values before treatment (lower *P* values indicated greater improvement in the expression of inflammatory mediators).

**Table 4:** Levels of IL-8, TNF-*α*, IL-17, and IL-23 in the blood of the LHQW group, the conventional group, and subgroups before and after treatment.

		Total		High-risk subgroups		Low-risk subgroups	
		LHQW group (*n* = 50)	Conventional group (*n* = 50)	LHQW group (*n* = 25)	Conventional group (*n* = 30)	LHQW group (*n* = 25)	Conventional group (*n* = 20)
IL-8	Before treatment (mean ± SD, pg/mL)	21.93 ± 7.56	20.67 ± 9.35	23.30 ± 8.29	21.25 ± 10.48	20.55 ± 6.65	19.78 ± 7.51
	After treatment (mean ± SD, pg/mL)	18.30 ± 6.55*	19.79 ± 7.87	19.74 ± 6.78	19.57 ± 8.00	18.41 ± 6.70*	16.32 ± 5.89
	*P* value	0.021	0.125	0.145	0.448	0.049	0.098

TNF-*α*	Before treatment (mean ± SD, pg/mL)	71.59 ± 23.30	72.52 ± 23.55	73.17 ± 23.95	73.88 ± 22.15	70.02 ± 23.01	70.48 ± 25.96
	After treatment (mean ± SD, pg/mL)	66.12 ± 21.46	67.33 ± 24.03	69.25 ± 23.61	66.87 ± 23.08	62.99 ± 19.06	68.01 ± 25.99
	*P* value	0.238	0.263	0.551	0.244	0.291	0.739

IL-17	Before treatment (mean ± SD, pg/mL)	111.62 ± 38.09	109.17 ± 29.07	116.53 ± 36.44	113.53 ± 32.64	106.71 ± 39.79	102.63 ± 21.89
	After treatment (mean ± SD, pg/mL)	93.16 ± 29.14**	101.49 ± 30.97	97.77 ± 26.06*	105.82 ± 31.97	88.56 ± 31.79*	94.99 ± 28.97
	*P* value	0.004	0.232	0.041	0.354	0.047	0.450

IL-23	Before treatment (mean ± SD, pg/mL)	68.55 ± 25.23	68.89 ± 28.29	72.98 ± 23.91	68.29 ± 30.59	64.12 ± 26.21	69.79 ± 25.20
	After treatment (mean ± SD, pg/mL)	61.59 ± 28.09	63.21 ± 28.24	68.79 ± 31.39	63.88 ± 30.67	54.39 ± 24.98	62.20 ± 24.88
	*P* value	0.208	0.303	0.617	0.563	0.169	0.335

SD: standard deviation, *P < 0.05 compared with values before treatment, **P < 0.01 compared with values before treatment (lower *P* values indicated greater improvement in the expression of inflammatory mediators).
